This article has been retracted.

# Distribution Characteristics of ST-Segment Elevation Myocardial Infarction and Non-ST-Segment Elevation Myocardial Infarction Culprit Lesion in Acute Myocardial Infarction Patients Based on Coronary Angiography Diagnosis

**DOI:** 10.1155/2022/2420586

**Published:** 2022-02-02

**Authors:** Guanglin Cao, Zheng Zhao, Zesheng Xu

**Affiliations:** ^1^Department of Cardiovascular Disease, Cangzhou Central Hospital of Tianjin Medical University, Tianjin 300000, China; ^2^Department of Cardiovascular Disease, First Central Clinical College of Tianjin Medical University, Tianjin 300000, China; ^3^Department of Cardiology, Tianjin First Central Hospital, Tianjin 300000, China

## Abstract

This research was aimed at exploring the application value of coronary angiography (CAG) based on a convolutional neural network algorithm in analyzing the distribution characteristics of ST-segment elevation myocardial infarction (STEMI) and non-ST-segment elevation myocardial infarction (NSTEMI) culprit lesions in acute myocardial infarction (AMI) patients. *Methods*. Patients with AMI treated in hospital from June 2019 to December 2020 were selected as subjects. According to the results of an echocardiogram, the patients were divided into the STEMI group (44 cases) and the NSTEMI group (36 cases). All patients received CAG. All images were denoised and edge detected by a convolutional neural network algorithm. Then, the number of diseased vessels, the location of diseased vessels, and the degree of stenosis of diseased vessels in the two groups were compared and analyzed. *Results*. The number of patients with complete occlusion (3 cases vs. 12 cases) and collateral circulation (5 cases vs. 20 cases) in the NSTEMI group was significantly higher than that in the STEMI group, and the difference was statistically significant, *P* < 0.05. There was a statistically significant difference in the number of lesions between the distal LAD (1 case vs. 10 cases) and the distal LCX (4 cases vs. 11 cases), *P* < 0.05. There was a statistically significant difference in the number of patients with one lesion branch (1 vs. 18) and three lesion branches (25 vs. 12) between the two groups, *P* < 0.05. The image quality after the convolution neural network algorithm is significantly improved, and the lesion is more prominent. *Conclusion*. The convolutional neural network algorithm has good performance in DSA image processing of AMI patients. STEMI and NSTEMI as the starting point of AMI disease analysis to determine the treatment plan have high clinical application value. This work provided reference and basis for the application of the convolutional neural network algorithm and CAG in the analysis of the distribution characteristics of STEMI and NSTEMI culprit lesions in AMI patients.

## 1. Introduction

Cardiovascular disease has always been the primary cause threatening the life and health of people in developed countries, and it will also become the main cause of death in developing countries in the future. Therefore, its diagnosis and treatment have gradually become the focus of research and attention [1–3]. Coronary atherosclerotic heart (CAD) disease causes a range of clinical manifestations. Common types include angina pectoris, acute coronary syndrome (ACS), arrhythmia, and even sudden cardiac death [4–6]. Acute myocardial infarction (AMI) is one of the most serious cases in the development of coronary heart disease, which poses a great threat to the life and health of patients [7]. At present, the main treatment principle for cardiovascular disease is to repair the damaged myocardium and quickly restore the blood supply to the heart. Therefore, accurate diagnosis of AML at an early stage is very important for diagnosis and treatment. Clinical studies showed that AMI can be divided into ST-segment elevation myocardial infarction (STEMI) and non-ST-segment elevation myocardial infarction (NSTEMI) according to ST-segment elevation [8]. ST-segment depression and no offset of NSTEMI electrocardiogram (ECG) are objective, and the risk of death is different in the two types of patients [9]. At present, the most effective method for the diagnosis of cardiovascular diseases is coronary angiography (CAG), which is regarded as the gold standard for the diagnosis of coronary artery diseases [10]. However, it takes a long time from the onset of AMI to the time of first medical contact and then to the opening of blood vessels, so the implementation of CAG requires corresponding equipment and professional operation [11, 12].

In recent years, the rapid development of artificial intelligence and big data has gradually penetrated into the medical field. How to extract effective features from massive medical images to provide basis for clinical disease diagnosis and treatment has become the focus of current research. Traditional learning algorithms are limited in feature extraction of medical images due to their weak feature expression ability caused by the shallow level of the training model. A depth learning algorithm is proposed under the background of advanced CPU, continuous improvement of machine algorithm, and massive medical images, which makes up for the defects of a traditional learning algorithm [13]. A large number of research data show that a supervised deep-learning algorithm has a good application effect in the field of image analysis. In particular, a deep convolutional neural network algorithm is a method with the most research value and potential in the field of image processing and analysis [14]. At present, there are many researches on the application of convolutional neural network in the field of medical image, and the common applications are image segmentation, image classification, image registration, and target detection [15]. Compared with other deep learning algorithms, the convolutional neural network algorithm has a convolutional layer that can be directly manipulated with two-dimensional data, so it has less robustness, and its error recognition rate is less than 0.1%. However, due to the complexity and low resolution of medical imaging, the convolutional neural network model needs to be further optimized. To address the above problems, a method was proposed in this research for image classification based on the existing convolutional neural network model, which had little difference in accuracy but can effectively reduce the parameter scale of the network. A complex convolutional neural network that shortens the training time of the network was put forward, and various parameter optimization works were performed on it.

In this study, STEMI and NSTEMI patients were selected as the research objects, and their CAG and echocardiogram were processed by convolutional neural network technology, and the imaging characteristics of patients were analyzed on this basis, in order to provide reference and basis for early clinical diagnosis of AMI patients.

## 2. Materials and Methods

### 2.1. Research Objects

Eighty patients with non-ST-segment elevation AMI who were treated in hospital from June 2019 to December 2020 were selected as the subjects. There were 60 males and 20 females, aged 37-88 years old, with an average age of 60.33 ± 11.6 years old. Inclusion criteria: (1) patients' persistent ischemic chest pain time more than half an hour, sublingual nitrate drugs, but chest pain does not relieve. (2) As time goes on, TnI or TnT is at least twice the maximum. (3) ECG showed ST-segment elevation less than l mv, ST-segment depression greater than or equal to 0.05 mv, or T wave inversion. (4) All patients underwent emergency interventional treatment within 72 h of onset. (5) All patients have complete medical records without missing important inspection items. Exclusion criteria: (1) old myocardial infarction, left main coronary artery disease, and ST-segment elevation AMI patients; (2) patients with other serious heart diseases such as rheumatic heart disease and primary cardiomyopathy; (3) patients cannot be performed CAG; (4) incomplete patient information; and (5) patients with AMI onset more than 72 h.

The selected patients were divided into the STEMI group (44 cases) and the NSTEMI group (36 cases) according to whether ST-segment of body surface ECG was depressed. STEMI diagnostic criteria: chest pain combined with troponin concentration or creatine kinase isoenzyme concentration exceeded the normal value, and ECG showed ST-segment arch upward elevation and had one or more of the following cases: persistent ischemic chest pain, an echocardiogram showing abnormal segmental wall motion, and abnormal CAG. NSTEMI diagnostic criteria: chest pain with troponin concentration or creatine kinase isoenzyme concentration exceeding the normal value and had one or more of the following cases: persistent ischemic chest pain, ECG showing new ST-segment depression, an echocardiogram showing abnormal segmental wall motion, and abnormal CAG. This study had been approved by the ethics committee of hospital, and all patients had signed the informed consent forms.

### 2.2. Inspection Method

The digital electrocardiograph was used to record the patient's 18-lead electrocardiogram in the supine position and calm breathing. 18-lead ECG were performed within 10 minutes of admission, once every 4-8 hours on the first day and once every 12-24 hours on the second day, for a total of 3 days. Interpretation analysis was conducted by two professional physicians, and the results of CAG were not informed to the analyst before ECG analysis. If the two judgment results are the same or close, they will be included, and if the difference is large, they will not be included. The ECG with the most significant changes in ST-segment was selected, and the TP-segment of each lead was observed first, and the equipotential line was set. The starting point of the QRS wave group was set as the ST-segment measurement base point (point J), the point 80 ms after point J was used as the standard point of ST-segment measurement, and the range of ST-segment offset was measured (measured by small grids of elevation/depression, if less than half grid, it was abandoned, and if more than half grid but less than one grid, it was counted as one grid), and six ST-segments were measured continuously. The mean value of the six measurements was taken as the ST-segment change value.

CAG process and IRA determination: CAG was interpreted by two associate chief physicians engaged in cardiology interventional direction, and the results were interpreted by superior chief physicians in case of disagreement. The RSITJUN method was used, digital subtraction angiography (DSA) was used to search for the coronary artery opening and merge path by traversing the brachial trunk to the aortic arch via the radial (or femoral) path. Conventional multiposition projection (right coronary artery projection 3 positions—left anterior oblique position, right anterior oblique position, left anterior oblique plus head position, left coronary artery projection 6 positions—left anterior oblique position, left anterior oblique plus head position, left anterior oblique plus foot position, right anterior oblique position, right anterior oblique plus head position, right anterior oblique plus foot position) was taken for selective left and right CAG to determine the location of coronary artery lesions, which were recorded as left anterior descending (LAD) branch, circumflex branch, and right coronary artery. The lesions involving one branch were recorded as single-branch lesions, involving two branches as double-branch lesions and involving three or more branches as multiple-branch lesions. If there were multiple-branch lesions, the most severe stenosis and thrombosis arteries were identified as infarct-related arteries (IRA criteria were thrombosis, residual stenosis, or spastic occlusion in the lumen). If the infarct-related artery spontaneously recanalization, its most narrow location is occlusion. In the process of angiography, the occlusion of the infarct-related artery can be judged by the following indirect signs: local filling of stenosis, defect signs, local contrast retention of stenosis, etc. Finally, the quantitative coronary analysis (QCA) system was used to accurately measure IRA, calculate the degree of vascular stenosis, and record TIMI blood flow classification and TIMI myocardial perfusion classification.

### 2.3. Image Processing Algorithm

Denoising processing: the array of image *f* (*x*, *y*) is *M* × *N*, the processed image is *g* (*x*, *y*), and its gray level is determined by the average gray level of several pixels in the field of (*x*, *y*). The processed image representation is as follows:

(1) $$\begin{array}{c} g\left(x,y\right)=\frac{1}{M}\underset{\left(i,j\right)\in s}{\sum }f\left(i,j\right). \end{array}$$

*x*, *y* = 0, 1, 2 ⋯ , *N* − 1, *S* is the domain set centered on (*x*, *y*) points, and *M* is the total number of coordinate points in *S*.

For multiple images, if the original image is *f* (*x*, *y*) and the noise is *n* (*x*, *y*), then the noise image *g* (*x*, *y*) is as follows:

(2) $$\begin{array}{c} g\left(x,y\right)=f\left(x,y\right)+n\left(x,y\right). \end{array}$$

The noise is uncorrelated, and the mean is zero.

(3) $$\begin{array}{c} f\left(x,y\right)=E\left[g\left(x,y\right)\right]. \end{array}$$

*E*[*g*(*x*, *y*)] is the expected value of *g*(*x*, *y*), and *M* noisy images are averaged.

(4) $$\begin{array}{c} f\left(x,y\right)=E\left[g\left(x,y\right)\right]\sim \bar{g}\left(x,y\right)=\frac{1}{M}\overset{M}{\underset{i=1}{\sum }}g_{i}\left(x,y\right), \end{array}$$

(5) $$\begin{array}{c} {\delta^{2}}_{\bar{g}\left(x,y\right)}={\delta^{2}}_{n\left(x,y\right)}, \end{array}$$

where ${\delta^{2}}_{\bar{g}\left(x,y\right)}$ and *δ*^2^_*n*(*x*, *y*)_ are the variances of $\bar{g}$ and *n* at point (*x*, *y*).

Edge detection is as follows:

(6) $$\begin{array}{c} \psi^{1}\left(x\right)=\frac{d\theta \left(x\right)}{dx},\\ \psi^{2}\left(x\right)=\frac{d^{2}\theta \left(x\right)}{dx^{2}}. \end{array}$$

### 2.4. Statistical Analysis

All data were analyzed by SPSS 19.0 statistical software. The measurement data were expressed by mean ± standard deviation. The test method was an independent sample *t*-test, and the comparison between groups depended on the chi-square test. The descriptive samples were tested by the independent sample nonparametric rank-sum Mann-Whitney *U* test. When *P* < 0.05, there was significant difference.

## 3. Results

### 3.1. General Data Comparison

The general data of the two groups were compared as shown in Table 1. Table 1 shows that a total of 80 patients were included in this study. The average age of the STEMI group was 63.11 ± 11.06. The average age of the NSTEMI group was 59.88 ± 11.76. There was no significant difference in age between the two groups, *P* > 0.05. There was no significant difference in the risk factors such as hypertension, hypercholesterolemia, diabetes, smoking history, and coronary heart disease history between the two groups, *P* > 0.05. It shows that the two groups of patients are comparable.

### 3.2. Display of Influence Data of Typical Cases

The images of classic cases before and after DSA angiography in the two groups are shown in Figure 1. CAG can clearly reflect the location and degree of coronary artery stenosis in patients. After the neural network algorithm, the image quality is significantly improved, the lesion is more prominent, and the details of the lesion are also well displayed.

### 3.3. Comparison of Coronary Stenosis Degree between the Two Groups

The comparison of the degree of coronary stenosis between the two groups is shown in Figure 2. According to the analysis of Figure 2, the number of patients with <50% in the STEMI group is 7, and the number of patients with narrowing degree between 50% and 74% is 11. The number of patients with narrowing degree between 75% and 99% is 22, the number of patients with complete occlusion is 3, and the number of patients with collateral circulation is 5. The number of patients with <50% in the NSTEMI group is 4, and the number of patients with narrowing degree between 50% and 74% is 5. The number of patients with narrowing degree between 75% and 99% is 11, the number of patients with complete occlusion is 13, and the number of patients with collateral circulation is 20. Comparing the number of patients with different degrees of stenosis between the two groups, it was found that the number of patients with complete occlusion (3 cases vs. 12 cases) and collateral circulation (5 cases vs. 20 cases) in the NSTEMI group was significantly higher than that in the STEMI group (*P* < 0.05). There was no significant difference in the number of patients with stenosis degree between 75%~99% and 50%~74% between the two groups (*P* > 0.05).

### 3.4. Comparison of Lesion Sites between the Two Groups

The comparison results of lesion sites between the two groups are shown in Figure 3. Figure 3 shows 9 cases of proximal LAD, 5 cases of middle LAD, and 1 case of distal LAD in the STEMI group. There were 5 proximal lesions, 9 middle lesions, and 5 distal lesions in RCA. There were 6 cases of proximal lesions and 4 cases of distal lesions in LCX. In LAD of the NSTEMI group, there were 2 cases of proximal lesions, 5 cases of middle lesions, and 10 cases of distal lesions. There were 2 cases of proximal lesions, 1 case of middle lesions, and 4 cases of distal lesions in RCA. There was 1 case of proximal lesions and 11 cases of distal lesions in LCX. There was significant difference between the two groups in the lesion location between the distal end of LAD (1 case vs. 10 cases) and the distal end of LCX (4 cases vs. 11 cases), *P* < 0.05.

### 3.5. Comparison of the Number of Diseased Coronary Arteries between the Two Groups

The comparison results of the number of coronary artery lesions in the two groups are shown in Figures 4 and 5. Figures 4 and 5 show that the number of coronary artery lesions in the STEMI group was 1 in 3 cases, 2 in 16 cases, and 3 in 25 cases. In the NSTEMI group, there were 18 cases with one coronary artery lesion, 6 cases with two coronary arteries, and 12 cases with three coronary arteries. There was a statistically significant difference in the number of patients with one lesion branch (1 vs. 18) and three lesion branches (25 vs. 12) between the two groups, *P* < 0.05.

## 4. Discussion

Coronary atherosclerotic heart disease (CHD), referred to as coronary heart disease, is one of the malignant diseases dangerous to human health [16]. ACS is one of the clinical types of coronary heart disease, which can be divided into three types: AMI, unstable angina pectoris, and sudden death [17]. AMI has the characteristics of high incidence rate, high mortality rate, acute onset, rapid change of state, and so on. According to echocardiographic results, it can be divided into two types: STEMI and NSTEMI [18]. When the intima is damaged, platelet exposure combined with the secretion of adhesion factors of endothelial cells leads to the aggregation of a large number of substances and the formation of white and transparent thrombus containing a large number of platelets. The thrombus makes the interior of the vascular lumen shrink rapidly or reach complete occlusion or subtotal occlusion through which a small amount of blood can pass [19]. Stress changes suddenly reduce the blood flow in the coronary artery, and the rapid contraction of blood vessels exacerbates pathological process. At this time, patients show unstable angina pectoris or non-ST-segment elevation [20]. If the thrombus is composed of fibrin network and a large number of red blood cells in the network, the red thrombus will completely block the lumen and stop the forward blood flow, which is manifested as ST-segment elevation myocardial infarction or sudden death [21, 22].

Different types of AMI have different characteristics, and treatment methods should also be different. The vascular lesions of NSTEMI are mainly multivessel lesions, with good short-term prognosis, high long-term mortality, and poor prognosis. The blood vessels of patients with NSTEMI are mostly incomplete occlusion lesions. The formation mechanism of collateral circulation is not clear. There are also many disputes in the treatment strategy and timing. Therefore, the understanding of AMI needs to be further improved [23]. For the diagnosis of AMI, CAG is still the gold standard for its diagnosis [24]. In recent years, CAG has been widely used in clinical practice, but there are also many shortcomings and limitations of this technology [25, 26]. In recent years, ultrasonic technology has been rapidly developed. Compared with CAG, it has the advantages of low cost, simple operation, and easy repetition. However, an echocardiogram also has some limitations, such as its diagnostic accuracy for cardiovascular diseases with complex conditions of multivessel disease is not high [27].

In recent years, the Internet and information technology have flourished. The corresponding various image processing technologies have also been rapidly developed, and medical image processing technology is one of the hot and key of research [28]. The deep convolution neural network algorithm is one of the most valuable and potential methods in the field of image processing and analysis. In the field of medical imaging, it is mainly used for the segmentation of lesions or the establishment of prognosis models of some tumors and cerebral hemorrhage, but it is rarely used in the field of cardiac diseases [29, 30]. In this study, the imaging data of different types of AMI patients such as DSA were studied on the basis of image processing by a convolution neural network algorithm. It is found that the quality of DSA image processed by a convolution neural network algorithm is more prominent. The most STEMI patients are coronary artery stenosis of 50%-74% and 75%-99%. Patients in the NSTEMI group had the most coronary artery stenosis with complete occlusion and collateral circulation. The lesions of the STEMI group were mostly concentrated in the proximal LAD and middle RCA. The lesions of the NSTEMI group were mostly concentrated in the distal LAD and distal LCX. The number of diseased coronary arteries in the STEMI group was two and three. The number of diseased coronary arteries in the NSTEMI group was mostly 1. In summary, the digital silhouette technology based on the convolutional neural network algorithm had a good effect and application value on the distribution characteristics of STEMI and NSTEMI culprit lesions in AMI patients. This was consistent with the conclusions of previous related studies.

## 5. Conclusion

In this study, the imaging data of different types of AMI patients such as DSA were studied on the basis of a convolution neural network algorithm. The number of patients with complete occlusion (3 cases vs. 12 cases) and collateral circulation (5 cases vs. 20 cases) in the NSTEMI group was significantly higher than that in the STEMI group, with statistical significance (*P* < 0.05). There was statistical difference in the number of lesions in distal LAD (1 case vs. 10 cases) and distal LCX (4 cases vs. 11 cases) between the two groups, *P* < 0.05. There was statistically significant difference in the number of coronary artery lesions between the two groups with 1 (1 vs. 18) and 3 (25 vs. 12), *P* < 0.05. This indicated that STEMI and NSTEMI as the entry point for diagnosis and analysis of disease had high clinical application value. The convolutional neural network algorithm shows better performance in DSA image processing of AMI patients. This study provides a reference and basis for clinical diagnosis of AMI. However, due to the limited samples, this study is not comprehensive and in-depth enough. In future study and work, it will be further expanded to continue to study this issue.

## Figures and Tables

**Figure 1:** DSA image display of typical cases.

**Figure 2:** Statistical results of coronary artery disease stenosis in the two groups. Note: compared with the STEMI group, ^∗^*P* < 0.05.

**Figure 3:** Statistical results of the lesions of the two groups of patients. Note: compared with the STEMI group, ^∗^*P* < 0.05.

**Figure 4:** Statistical results of the number of coronary artery lesions in the STEMI group.

**Figure 5:** Statistical results of the number of coronary artery lesions in the NSTEMI group.

**Table 1:** Comparison of general data of two groups of patients.

Item	STEMI	NSTEMI	*P*
	*n* = 44	*n* = 36	
Age (years)	63.11 ± 11.06	59.88 ± 11.76	0.07
Hypertension (%)	53.88	55.9	0.32
Diabetes (%)	49.8	39.9	0.13
Smoking (%)	27.81	32.1	0.18
Heart rate (beat/min)	77.73 ± 10.22	68.03 ± 10.16	0.13
Systolic pressure (mmHg)	137.02 ± 18.31	136.14 ± 17.94	0.09
Diastolic blood pressure (mmHg)	85.07 ± 14.44	86.28 ± 9.66	0.14
White blood cells (×10^9^)	8.53 ± 2.17	8.65 ± 2.09	0.13
Low density lipoprotein (mmol/L)	2.43 ± 0.81	2.64 ± 0.53	0.15
Triglyceride (mmol/L)	1.39 ± 0.46	1.48 ± 0.68	0.12
Fibrinogen (g/L)	2.83 ± 0.54	3.09 ± 0.71	0.13
Blood glucose (mmol/L)	9.11 ± 3.93	9.06 ± 4.43	0.23
CK-MB (U/L)	85.83 ± 20.15	84.09 ± 18.36	0.33
cTnT (ng/L)	1.36 ± 0.81	0.83 ± 0.68	0.069
NT-proBNP	1925.81 ± 2284.3	1918.84 ± 1147.2	0.38
EF (%)	55.66 ± 8.33	57.68 ± 9.33	0.33
Left ventricular end diastolic diameter (mm)	45.7 ± 3.77	49.35 ± 4.47	0.51

## Data Availability

The data used to support the findings of this study are available from the corresponding author upon request.
